# Hyperbaric Oxygen Improves the Survival and Angiogenesis of Fat Grafts after Autologous Fat Transplantation

**DOI:** 10.1155/2022/6738959

**Published:** 2022-05-20

**Authors:** Fei Liu, Zhi Liang, Ye Cui, HaiBo Lin, ZhengDong Guo, WangChi Qin, Bin Cheng, WeiGuo Yang

**Affiliations:** Department of Plastic and Cosmetic Surgery, Huazhong University of Science and Technology Union Shenzhen Hospital, Shenzhen, 518052 Guangdong, China

## Abstract

**Objective:**

Currently, autologous fat transplantation (AFT) still has a low graft survival rate. Elevation of the AFT graft survival rate is a challenge. This study investigated the effect of hyperbaric oxygen (HBO) on AFT.

**Methods:**

Twelve adult male SD rats were randomly divided into two groups after AFT: the control group (*n* = 6) and the HBO group (*n* = 6). The rats were killed at 7, 14, and 28 days after transplantation to take the transplanted adipose tissues. The volume and weight of the tissues were detected. The pathological changes in the adipose tissues were observed after H&E staining. Microvessel density and levels of transforming growth factor- (TGF-) *β*, tumor necrosis factor- (TNF-) *α*, and malondialdehyde (MDA) in the transplanted adipose tissues were measured with CD31 immunohistochemical stain, ELISA, and biochemical reagents, respectively. Additionally, the protein expression levels of vascular endothelial growth factor- (VEGF-) A and platelet-derived growth factor- (PDGF) A in the adipose tissues were detected by Western blot.

**Results:**

HBO significantly preserved the volume and weight of the transplanted adipose tissue (*p* < 0.01) and maintained the pathological structure of the transplanted adipose tissue. HBO therapy was effective in reducing inflammatory factor (TGF-*β* and TNF-*α*) levels and oxidative stress (MDA) in the transplanted adipose tissue (*p* < 0.01) and significantly increased the level of CD31 and angiogenesis-related factors including VEGF-A and PDGF-A (*p* < 0.01) to promote angiogenesis.

**Conclusion:**

HBO therapy regulated the immune response of fat grafts, stimulated their angiogenesis, and ultimately promoted their survival after AFT.

## 1. Introduction

Autologous fat transplantation (AFT) is a process in which fat is obtained from a part of the body and injected into the other areas that required treatment [1]. Adipose tissue is abundant in most human bodies and is readily accessible by liposuction. AFT has been proven safe when used for aesthetic purposes [2] and has become an established method in plastic surgery over the past three decades [3]. Caviggioli et al. found that AFT was an effective, safe, relatively noninvasive, and rapid surgical method for postmastectomy pain syndrome [4]. Maione et al. confirmed AFT was a safe treatment with a low complication rate, and its effect in treating Achilles tendon region wounds depended on the biological characteristics of adipose tissue. These characteristics were quite evident in reepithelialization of chronic ulcers and the enhancement of softness of perilesional tissue [5]. Zhao et al. demonstrated that in the treatment of the Parry-Romberg syndrome, AFT was conducive to the recovery of facial contour and symmetry in patients [6]. In addition, there were also many other studies pointing out that AFT could be promising in the treatment of neuropathic pain such as pain from scars [7, 8].

Autologous fat has been proven as an ideal material for soft tissue augmentation due to its biocompatibility, versatility, naturalness, nonimmunogenicity, inexpensiveness, and easy availability as well as the low disease incidence at the donor site [9]. However, at present, the main obstacle in the application of AFT is its uncontrollable and low graft survival rate and its absorption rates ranging between 25% and 80% [10]. Therefore, there is an urgent need to find ways to increase the graft survival rate. Sufficient neovascularization in the transplanted fat is necessary for the survival and long-term maintenance of grafts [11], so the following researches should be focused on promoting neovascularization at the recipient site after AFT.

AFT currently still induces some complications, including calcification, oil cysts, and fat necrosis. And adipokines released from transplanted white adipose tissue may contribute to the development of chronic inflammation [12]. Procurement, cell processing, transplantation, and recipient site management are referred to as the primary procedures of AFT [13]. Each step can affect graft volume retention, and this effect is thought to be caused by a cascade of mechanical injury, ischemia/hypoxic injury, and oxidative stress [14, 15]. It has therefore been pointed out that the prevention of oxidative stress during liposuction deserves in-depth discussion.

Hyperbaric oxygen (HBO) therapy is a new treatment during which patients are placed in a pure O_2_ pressurized chamber with 2.0-3.0 atmospheric absolute pressure [16]. For different conditions, the treatment can last from about 1.5 to 2 hours and be performed 1 to 3 times per day [16]. At present, HBO therapy is widely used in clinical practices, and it is effective in the treatment of a variety of diseases. For example, HBO accelerates wound healing and reduces the risk of amputation when used as an adjunct to treat refractory diabetic lower extremity wounds and delayed radiation injury [17]. It can reduce coronary restenosis after balloon angioplasty/stenting [18] and prevent muscle loss that occurs after thrombolytic therapy for myocardial infarction [19]. In liver transplantation surgery, HBO therapy can restore the liver function of donors more rapidly and improve the liver survival rate of receptors [20]. Studies have also shown that HBO therapy can significantly contribute to the success of limb implantation and free tissue transfer [21]. Feldmeier et al. have reported that HBO therapy can serve as an effective adjuvant therapy to increase skin graft and flap survival [22]. Collectively, HBO therapy not only plays a pivotal role in the treatment of diseases but also contributes to the success rate of organ transplantation. Following this idea, we hypothesized that HOB could improve the graft survival in FAT and explored the improving effect of HOB on the transplanted adipose tissue survival in a FAT rat model. This study may provide a directional reference and data basis for promoting the survival rate of clinical fat transplantation.

## 2. Materials and Methods

### 2.1. Experimental Animals

Twelve SPF adult male SD rats weighing 220 ± 30 g were housed at 22°C and 60% relative humidity (RH) in a 12/12 h dark/light environment and fed ad libitum. Subsequent experiments were conducted after adaptive feeding for 7 days. This study was approved by the Experimental Animal Ethics Committee of Guangdong Medical Experimental Center (C202203-29).

### 2.2. Construction of a Rat Model for Autologous Fat Transplantation

The rats were anesthetized. A 2.5 cm incision was made on the inguinal fold to obtain an inguinal fat pad of about 50 mg. Subsequently, a 1 cm incision was made on the dorsal surface of the scapula, and the fat pad was cut into small pieces and placed in the incision. Finally, the wound was closed. After that, the rats were randomly divided into two groups. In the control group (*n* = 6), rats received no other treatment after surgery. In the HBO group, rats were placed in a pressurized chamber, with a compression time of 10 min at 2.0 atmospheric absolute pressure. The rats breathed 100% oxygen, with a maintaining time of 60 at 2.0 atmospheric absolute pressure and a decompression time of 5 min. According to the above treatment regimen, rats received HBO treatment once a day and were killed at 7, 14, and 28 days after transplantation to collect the transplanted adipose tissues [23].

### 2.3. H&E Staining

Detecting the tissue was fixed in 4% paraformaldehyde, embedded, sectioned, and fixed on a glass slide. Following, the slide was stained with hematoxylin differentiated with hydrochloric acid alcohol and bluing with 1% ammonia, rinsed with water, and then stained with eosin for 30 s. Prior to mounting, the sample was dehydrolized with alcohol and cleaned with xylene. Finally, a biological microscope was employed to observe the tissue and obtain images.

### 2.4. ELISA

TGF-*β* and TNF-*α* in the adipose tissue were detected with ELISA kits (Multisciences (Lianke) Biotech, Co., Ltd., China) by following the product instructions.

### 2.5. Malondialdehyde Detection

The level of malondialdehyde (MDA) in tissues was detected as per the instructions of the MDA kit (Beyotime, Shanghai, China).

### 2.6. Immunohistochemical Detection

Detecting transplanted adipose tissue was fixed with 4% paraformaldehyde for 48 h, embedded, and sectioned with a slice thickness of 4 *μ*m. The sections on a glass slide were then soaked in 100%, 95%, 85%, and 75% alcohol rinsed with double-distilled water, blocked with serum in PBST buffer, and coincubated with the primary antibody overnight. After washing with PBST buffer, the sections were reacted with enzyme-labeled secondary antibodies for 60 min again and finally mounted. The results were observed with a microscope, and the microvessel density was quantified.

### 2.7. Western Blot

20 *μ*g of the protein extracted from the detecting tissue was denatured by boiling, separated in a SDS-PAGE, and transferred on PVDF membranes. After blocking with 5% nonfat dry milk powder, the membrane was reacted with primary antibodies overnight, washed three times, incubated with secondary antibodies for one hour at room temperature, washed again in triplicate, and developed by adding chemiluminescence reagent to visualize the probed proteins. Densitometry of the protein bands was analyzed with the ImageJ software. The relative protein expression was calculated with *β*-actin as an internal reference.

### 2.8. Statistical Analysis

SPSS 26.0 was employed for analysis. The data were expressed as mean ± standard deviation. The independent *t*-test was used for comparison between the two groups. One-way ANOVA analysis of variance was used for comparison among multiple groups. *p* < 0.05 was defined as a statistically significant difference.

## 3. Results

### 3.1. HBO Maintained the Structure of the Adipose Grafts

The effect of HBO on adipose grafts was first examined. The results showed that the volume and weight of the adipose tissues gradually decreased along with the given periods (7, 14, and 28 days) after transplantation in the control group (*p* < 0.01). However, this pattern did not significantly occur in the HBO group 7-28 days after transplantation (*p* > 0.05) (Figures 1(a) and 1(b)). According to H&E staining results, the control group showed extensive fibrosis, proliferation of peripheral fibrous tissue, necrosis of adipose tissue, and formation of vacuoles at 7, 14, and 28 days after transplantation. By contrast, the grafts in the HBO group performed better stability, and the number of vacuoles and occurrence of necrosis, inflammatory response, and fibrosis were significantly lower than those in the control group (*p* < 0.01) (Figure 1(c)).

### 3.2. HBO Significantly Reduced the Levels of Inflammatory Factors and Oxidative Stress in the Fat Grafts

The effects of HBO on the levels of inflammatory factors and oxidative stress in fat grafts were further examined. There was no significant difference in the levels of TGF-*β* and MDA in the grafts between the two groups at 7 days after transplantation; however, the level of TNF-*α* in the HBO group was significantly lower than that in the control group. At 14 and 28 days after transplantation, lower levels of TNF-*α* and MDA in the grafts were identified in the HBO group compared with the controls (*p* < 0.01). The level of TGF-*β* only significantly decreased at 28 days in the HBO group compared with that of the controls (*p* < 0.01). Thus, the levels of TGF-*β*, TNF-*α*, and MDA in the tissues of the two groups gradually decreased over time with a more significant decrease observed in the HBO group (Figure 2).

### 3.3. HBO Significantly Promoted Angiogenesis and Immune Regulator after Fat Transplantation

Further examination was conducted to figure out the promoting effect of HBO on angiogenesis after AFT. The vessels of the fat grafts were estimated by the CD31 immunochemical stain. The results implied that the levels of the CD31 and microvessel density in the adipose tissue in the HBO group were significantly higher than those in the control group on the 7th, 14th, and 28th days after transplantation (*p* < 0.01) (Figure 3(a)). Meanwhile, Western blot results also showed that the protein expression levels of proangiogenic factors and immune chemokine, including VEGF-A and PDGF-A, in the tissue of the HBO group were significantly higher than those in the control group at these three time points (*p* < 0.01) (Figure 3(b)).

## 4. Discussion

Improving the oxygenation of fat grafts is an approach to increase the activity of phagocytes and fibroblasts as well as promote collagen formation and angiogenesis [24]. Under HBO therapy, the patient has his entire body at a pressure above sea level to receive intermittent treatment with 100% oxygen. Such therapy can improve oxygen-related pathological and physiological conditions of the wounds and speed the healing process via increasing the oxygen in the arteries. With a deeper understanding of HBO therapy, it has been widely used as adjuvant therapy for various pathological conditions, mainly hypoxic and/or ischemic diseases including arterial gas embolism, carbon dioxide poisoning, soft tissue infection, and refractory osteomyelitis. The indications of HBO therapy continue to increase. HBO therapy has been shown to improve graft organ survival, such as liver transplantation [20], limb implantation and free tissue transfer [21], and skin graft and flap survival [22]. In another study, HBO therapy applied before skin grafting and three days after grafting could significantly improve graft survival by 29% [25]. Other studies have also reported that HBO can improve the integrity of transplanted adipose tissue [24]. These findings strongly hint that HBO therapy may play a positive role in the AFT. Based on this idea, we performed this study and found that HBO therapy lasting 28 days significantly improved the structure of fat grafts and remarkably increased their survival rate. Such treatment can increase body blood flow and oxygen supply [26]. Theoretically, HBO therapy can increase the oxygen required for oxidative phosphorylation in the mitochondria and contribute to the production of adenosine triphosphate and the viability of cells, thus exerting beneficial effects on graft retention and survival [27]. Additionally, the positive effect of HBO therapy on liver transplantation and preservation has been proved [28]. It is therefore clear that HBO therapy can increase the survival rate of fat grafts.

Inflammation crucially impacts allograft survival and acceptance. Oweira et al. reported that macrophage inflammatory protein 2 and TNF-*α* are abnormally increased in a study on skin allograft rejection [29]. Zhu et al. showed that the IGF-*β* application accelerates acute hepatic rejection [30]. It has been shown that edaravone combined with HBO therapy markedly reduces oxidative stress and inflammatory factor levels in patients with acute intracerebral hemorrhage [31]. Similarly, our study indicated that both IGF-*β* and TNF-*α* were significantly upregulated in the AFT rat. HBO application remarkably declined these elevations in the AFT rats. Oxidative stress activation plays an important role in the transplantation rejection [32]. Our data revealed that HBO treatment successfully declined the AFT-induced MDA elevation, suggesting that HBO has an antioxidative stress activity. The vascular net establishment is a basic process for grafted tissue survival. Proangiogenesis becomes a strategy to improve grafted tissue survival [33]. Interestingly, inflammation and oxidative stress in the tissues showed an improvement after HBO therapy in our study. Our study also found the positive effect of HBO therapy on the generation of angiogenesis-related factors and angiogenesis in the AFT rat model. According to previous studies, neovascularization occurs through two mechanisms. One is the sprouting of local endothelial cells (angiogenesis), and the other is the recruitment and differentiation of circulating stem/progenitor cells (vasculogenesis) [34]. HBO therapy affects both mechanisms. That means HBO therapy, on the one hand, can stimulate the body to produce a large amount of reactive oxygen species and directly stimulate the production of circulating stem/progenitor cells [35] and, on the other hand, acts to stimulate the transcription of many genes related to neovascularization by stabilizing hypoxia-inducible factor [36]. Based on the above findings, it can be concluded that HBO can improve the survival rate of grafts by increasing angiogenesis. Immunosuppression has always been the key to the success of organ transplantation. Our results showed that HBO therapy not only had anti-inflammatory, antioxidant stress, and proangiogenesis activities but also had a certain immunosuppressive effect (inhibiting PDGF-A activity).

## 5. Conclusions

HBO can significantly improve the grafted adipose tissue survival and success rate through the anti-inflammatory response, antioxidative stress, immunosuppression, and proangiogenesis activities. Therefore, HBO therapy is highly promising as an adjuvant treatment following fat transplantation in clinical practice. However, our experiments were conducted on rats only; further clinical trials are required to provide more accurate experimental data and a solid basis.

## Figures and Tables

**Figure 1:** Effect of hyperbaric oxygen on the adipose grafts. The average (a) volume and (b) weight of the adipose grafts in the HBO (blue) and control (red) groups were measured at the indicated time. (c) H&E stain showed the pathological structure of the adipose grafts in the rats of either the HBO (up panels or blue bars) or the control (low panels or red bars) at the indicated times. ^∗∗^*p* < 0.01 vs. the control group; ^##^*p* < 0.01 vs. day 7; ^&&^*p* < 0.01 vs. day 14.

**Figure 2:** Effect of HBO on TGF-*β*, TNF-*α*, and MDA levels in the fat grafts. The (a) TGF-*β*, (b) TNF-*α*, and (c) MDA levels of the adipose grafts in the rats of either the HBO (blue) or the control (red) at indicated times were analyzed by ELISA and/or biochemical analysis. ^∗∗^*p* < 0.01 vs. the control group; ^##^*p* < 0.01 vs. day 7; ^&&^*p* < 0.01 vs. day 14.

**Figure 3:** Effect of HBO on angiogenesis in the fat grafts. (a) The blood vessels of the HBO (right panel) and control (left panel) samples were estimated by the CD31 immunohistochemical staining in the fat grafts at indicated times. (b) The protein expression levels of VEGF-A and PDGF-A were detected by Western blot in the HBO (right panels or blue bars) and the control (left panels or red bars) groups of the fat grafts at indicated times. MVD: microvessel density. ^∗∗^*p* < 0.01 vs. control group.

## Data Availability

The data used to support the findings of this study are available from the corresponding author upon request.
